# Chotosan ameliorates cognitive and emotional deficits in an animal model of type 2 diabetes: possible involvement of cholinergic and VEGF/PDGF mechanisms in the brain

**DOI:** 10.1186/1472-6882-12-188

**Published:** 2012-10-20

**Authors:** Qi Zhao, Yimin Niu, Kinzo Matsumoto, Koichi Tsuneyama, Ken Tanaka, Takeshi Miyata, Takako Yokozawa

**Affiliations:** 1 Division of Medicinal Pharmacology, Institute of Natural Medicine, University of Toyama, 2630 Sugitani, 2630 Sugitani, Toyama 930-0194, Japan; 2 Department of Diagnostic Pathology, Graduate School of Medical and Pharmaceutical Sciences, University of Toyama, 2630 Sugitani, Toyama, 930-0194, Japan; 3 Division of Pharmacognosy, Institute of Natural Medicine, University of Toyama, 2630 Sugitani, Toyama, 930-0194, Japan; 4 Division of Biomedical Informatics, Institute of Natural Medicine, University of Toyama, 2630 Sugitani, Toyama, 930-0194, Japan; 5 Laboratory of Presymptomatic Medical Pharmacology, Faculty of Pharmaceutical Sciences, Sojo University, 4-22-1 Ikeda, Kumamoto, 860-0082, Japan; 6 Collaboration Division, Organization for Promotion of Regional Collaboration, University of Toyama, 3190 Gofuku, Toyama, 930-8555, Japan

**Keywords:** Chotosan, Diabetes, Cognitive deficits, Cholinergic system, VEGF/PDGF systems

## Abstract

**Background:**

Diabetes is one of the risk factors for cognitive deficits such as Alzheimer’s disease. To obtain a better understanding of the anti-dementia effect of chotosan (CTS), a Kampo formula, we investigated its effects on cognitive and emotional deficits of type 2 diabetic *db/db* mice and putative mechanism(s) underlying the effects.

**Methods:**

Seven-week-old *db/db* mice received daily administration of CTS (375 – 750 mg/kg, p.o.) and the reference drug tacrine (THA: 2.5 mg/kg, i.p.) during an experimental period of 7 weeks. From the age of 9-week-old, the animals underwent the novel object recognition test, the modified Y-maze test, and the water maze test to elucidate cognitive performance and the elevated plus maze test to elucidate anxiety-related behavior. After completing behavioral studies, Western blotting and immunohistochemical studies were conducted.

**Results:**

Compared with age-matched non-diabetic control strain (*m/m*) mice, *db/db* mice exhibited impaired cognitive performance and an increased level of anxiety. CTS ameliorated cognitive and emotional deficits of *db/db* mice, whereas THA improved only cognitive performance. The phosphorylated levels of Akt and PKCα in the hippocampus were significantly lower and higher, respectively, in *db/db* mice than in *m/m* mice. Expression levels of the hippocampal cholinergic marker proteins and the number of the septal cholinergic neurons were also reduced in *db/db* mice compared with those in *m/m* mice. Moreover, the *db/db* mice had significantly reduced levels of vasculogenesis/angiogenesis factors, vascular endothelial growth factor (VEGF), VEGF receptor type 2, platelet-derived growth factor-B, and PDGF receptor β, in the hippocampus. CTS and THA treatment reversed these neurochemical and histological alterations caused by diabetes.

**Conclusion:**

These results suggest that CTS ameliorates diabetes-induced cognitive deficits by protecting central cholinergic and VEGF/PDGF systems via Akt signaling pathway and that CTS exhibits the anxiolytic effect via neuronal mechanism(s) independent of cholinergic or VEGF/PDGF systems in db/db mice.

## Background

Diabetes is one of the most important risk factors implicated in cognitive deficits such as Alzheimer’s disease (AD) and vascular dementia (VD) and is associated with impaired cognitive function, including learning, memory, and processing speed [1,2]. In a previous clinical study, about 80% of AD patients appeared to be diabetic or to have abnormal blood glucose levels and defects in insulin signaling that were associated with accumulation of the neurofibrillary tangles (NFTs) and senile plaques of AD [3]. Similar learning and memory deficits have been demonstrated in *db/db* mice, an animal model of type 2 diabetes that fails to respond to leptin, a 16 kDa protein hormone with a key role in appetite, metabolism, and regulation of energy intake and energy expenditure [4,5]. This animal model exhibits not only hyperglycemia and hyperinsulinemia but also impaired cognitive performance, long-term potentiation, and emotional behavior [6]. These deficits have been reported to become evident in adulthood at 10 weeks old and over. However, the mechanisms underlying cognitive dysfunction in diabetes have not been clearly understood [3].

Chotosan (CTS, or Gouteng San in traditional Chinese medicine) is a Kampo (i.e. Chinese medicine) formula consisting of ten medicinal herbs and gypsum fibrosum. It has long been used to treat chronic headache, painful tension of the shoulders and cervical muscles, vertigo, morning headache, a heavy feeling of the head, flushing, tinnitus, and insomnia, particularly in middle-aged or older patients with weak physical constitutions [7]. Moreover, double-blind and placebo-controlled clinical studies [7,8] demonstrated that CTS is effective in the treatment of stroke patients with cognitive impairments and patients with mild to moderate dementia of the Alzheimer type [9]. Consistent with these clinical findings, it was demonstrated that daily administration of CTS improves cerebral flow and exhibits an anti-hypertensive effect in spontaneously hypertensive rats [10,11]. In addition, we reported that CTS ameliorates cognitive deficits observed in animal models of vascular dementia [12,13] and suggested that the effects of CTS are mediated by amelioration of dysfunction of central cholinergic systems, which play an important role in learning, memory, and cognitive performance. These clinical and neuropharmacological findings raise the possibility that not only central cholinergic systems but also factors/mechanism(s) involved in the blood circulation system may account for anti-dementia effects of CTS.

Evidence indicates that the angiogenic growth factors VEGF and PDGF are involved in the adverse vascular effects of hyperglycemia such as diabetic nephropathy and retinopathy [14,15]. However, retardation of angiogenesis, particularly in the brains of aged animals is severe enough to impair synaptic plasticity, a molecular biological process important in learning and memory, and requires long-lasting increases in metabolic demand supported by the generation of new capillaries [16]. Indeed, recent findings have indicated that VEGF and PDGF are important not only in angiogenesis but also in neuroprotection and neurogenesis in the brain [16] and that elevation of the levels of these factors improves cognitive and emotional performance in an animal model of dementia [17-21]. Moreover, in the peripheral system, the protective effect of cholinergic drugs such as donepezil, an acetylcholinesterase inhibitor against AD, on ischemic cell damage appears to be mediated by phosphatidyl inositol-3 phosphate kinase/Akt phosphorylation/VEGF systems. We have recently reported that CTS administration also exhibits a beneficial effect on cognitive deficits caused by aging, one of the risk factors for Alzheimer disease (AD) and cerebrovascular disease-related dementia [22] and that amelioration of VEGF/PDGF systems in the brain is likely involved in the effects of CTS [20]. These findings prompted us to investigate whether CTS can ameliorate diabetes-related neuropsychiatric symptoms and, if so, whether cholinergic and VEGF/PDGF systems are involved in the action of CTS in the *db/db* mice. For this aim, we used tacrine, an acetylcholinesterase inhibitor with anti-dementia activity, and compared its effects on diabetes-induced cognitive and emotional deficits and neurochemical alterations with those of CTS.

## Methods

### Animals

Male 6-week-old C57BLKS/J-*db/db* mice and their age-matched non-diabetic *m/m* littermates were purchased from Japan SLC Inc. (Hamamatsu, Japan). The animals were housed in groups of 6 – 9 mice/cage (24 × 17 × 12 cm) in a laboratory animal room, which are maintained at 25 ± 1°C with 65 ± 5% humidity, on a 12 h light/dark cycle (lights on: 07:30-19:30) for 1 week before the start of the experiments. The animals were given food and water *ad libitum*. The study was conducted according to the experimental schedule depicted in Figure 1. After 1 week of acclimatization, blood samples were collected from the tail vein to measure serum glucose level. The *db/db* mice were randomly divided into 5 groups and then received daily administration of the test drugs, except for one group that was used for anxiolytic drug treatment. The drug administration was continued during the experimental period. All animal research procedures used in the present study were in accordance with the Guiding Principles for the Care and Use of Animals (NIH Publications No. 80-23, revised in 1996). The present study was also approved by the Institutional Animal Use and Care Committee of the University of Toyama (approval No.: S-2009 INM-1).

**Figure 1:** **Schematic drawing of experimental schedule.** After one week of acclimatization, the *db/db* mice were randomly divided into 5 groups. Age-matched *m/m* and *db/db* mice were used as controls in the behavioral and neurochemical experiments.

### Drug treatment

Test drug administration was performed using a feeding needle once daily at around 9 a.m. during the experimental period. The *m/m* and *db/db* vehicle (control) groups were given water perorally (p.o.), while the other groups were orally administered CTS daily at doses of 375 and 750 mg/kg body weight or injected intraperitoneally with THA (2.5 mg/kg) (Sigma-Aldrich Japan, Tokyo, Japan) dissolved in physiological saline, except when stated otherwise.

### Preparation and chemical profiling of CTS extract

CTS used in this study was purchased from Tsumura Co. (Tokyo, Japan) and was the same lot (Lot #202004-7010) as used in previous studies [13,20]. CTS was extracted from a mixture of 3.0 parts *Uncariae Uncis cum Ramulus* (hooks and branch of *Uncaria rhynchophylla* MIQUEL), 3.0 parts *Aurantii Nobilis pericarpium* (peel of *Citrus unshiu* MARKOVICH), 3.0 parts *Pinelliae tube*r (tuber of *Pinellia ternate* BREITENBACH), 3.0 parts Ophiopogonis tuber (root of *Ophiopogon japonicus* KER-GAWLER), 3.0 parts Hoelen (sclerotium of *Poria cocos* WOLF), 2.0 parts Ginseng radix (root of *Panax ginseng* C.A. MEYER), 2.0 parts Saphoshnikoviae radix (root and rhizome of *Saposhnikovia divaricata* SCHISCHKIN), 2.0 parts Chrysanthemi flos (flower of *Chrysanthemum morifolium* RAMATULLE), 1.0 part Glycyrrhizae radix (root of *Glycyrrhiza uralensis* FISHER), 1.0 part Zingiberis rhizome (rhizome of *Zingiber officinale* ROSCOE), and 5.0 parts Gypsum fibrosum (CaSO_4_ 2H_2_O). The yield of CTS extract was 16.1%. To identify the chemical constituents of CTS, 3 dimensional high-performance liquid chromatography (3D-HPLC) analysis was conducted as previously described [11,13]. Briefly, Chotosan (2.5 g, Tsumura, Tokyo, Japan) was filtered and then subjected to HPLC analysis. HPLC equipment was controlled with an SLC-10A (Shimadzu, Kyoto, Japan) using a TSKGELODS-80TS column (4.6 × 250 mm), eluting with solvents (A) 0.05 M AcONH_4_ (pH 3.6) and (B) CH_3_CN. A linear gradient of 100% A and 0% B changing over 60 min to 0% A and 100% B was used. The flow rate was controlled with an LC-10 AD pump at 1.0 ml/min. The eluent from the column was monitored and was processed using an SPD-M10A diode array. For chemical profiling of CTS, liquid chromatography-mass spectrometry (LC-MS) analysis was performed with a Shimadzu LC-IT-TOF mass spectrometer equipped with an electrospray ionization (ESI) interface. The ESI parameters were as follows: source voltage +4.5 kV, capillary temperature 200°C, and nebulizer gas 1.5 l/min. The mass spectrometer was operated in positive ion mode scanning from *m/z* 200 to 2000. A Waters Atlantis T_3_ column (2.1 mm i.d. × 150 mm, 3 μm) was used and the column temperature was maintained at 40°C. The mobile phase was a binary eluent of (A) 5 mM ammonium acetate solution and (B) CH_3_CN under the following gradient conditions: 0-30 min linear gradient from 10% to 100% B, 30-40 min isocratic at 100% B. The flow rate was 0.15 ml/min. Mass spectrometry data obtained from the extract have been listed in MassBank database [23] and stored together with the pharmacological information on the extract in the Wakan-Yaku Database system (WakanDB ID: LCMS: Chotosan/11000001 http://wakandb.u-toyama.ac.jp/wiki/LCMS:Chotosan/11000001), Institute of Natural Medicine, University of Toyama. Voucher specimen (CTS: No. 2020047010) obtained from Tsumura Co. Ltd. has been deposited at our institute.

### Measurement of serum glucose

Before and after completing the behavioral studies, serum samples were collected from tail vein of each animal group under pentobarbital (50 mg/kg, i.p.) anesthesia. The serum glucose levels were measured using a commercially available kit (Glucose CII-Test, Wako Pure Chem., Osaka, Japan) as previously described [5].

### Behavioral assessment

#### Novel object recognition test (ORT)

ORT was conducted as previously described [13,20,21]. The apparatus consisted of a square arena (50 × 50 × 40 cm) made of polyvinyl chloride with gray walls and a black floor (Figure 2A). The objects for recognition had visual patterns or visually different shapes to enable discrimination. The ORT consisted of a sample phase trial and a test phase trial. In the sample phase trial, each mouse was first placed in the observation box where two identical objects, objects O1 and O2 (each of which was a 7.5 × 5.5 cm white cup), were placed separately, and allowed to explore the arena freely for 10 min. The total time that the mouse spent exploring each of the two objects was measured and then the mouse was returned to the home cage. In the test phase trial performed 30 min after the sample phase trial, one of the two objects was replaced by an identical copy (object F) and the other by a novel object (object N). Performance of the animals in this test was video-recorded for later analysis. In these trials, the exploration of an object was defined as directing the nose to the object at a distance of <2 cm according to previous reports [13,21,24] and the time spent exploring each of the two objects was analyzed using SMART® ver. 2.5 (PanLab, S.L., Barcelona, Spain) with a tri-wise module to detect the head, center mass, and base-tail. A discrimination index (DI) was calculated according to the following equation [13,21,24]: DI = (T_n_ − T_f_)/(T_n_ + T_f_). Here, T_n_ and T_f_ represent the times spent exploring new and familiar objects, respectively. The box arena and objects were cleaned using 75% ethanol between trials to prevent a build-up of olfactory cues.

**Figure 2:** **Effects of CTS and THA on object discrimination performance of *db/db *mice in the ORT.** The ORT was conducted on days 19–21 after starting drug administration. Each datum represents the mean ± S.D. (6 – 9 mice per group). (**A**) The data from the sample trials of the ORT. The animal was placed into the arena where two identical sample objects made of glass (objects A1 and A2) were placed in two adjacent corners of the arena and was allowed to explore for five minutes. (**B**) The data from the test phase trials conducted ten minutes after the sample phase trials. In the test phase trials, the time animals spent exploring a familiar object or a new object was measured during a 5-minute observation period. ***P < 0.001 and **P < 0.01 vs. the time spent exploring a familiar object (paired *t*-test). (**C**) Discrimination index (DI) in the ORT. DI was calculated as described in the text. **P < =0.01 vs. vehicle-treated *m/m* group (*t*-test). *P < 0.05 vs. vehicle-treated *db/db* group Tukey test.

#### Modified Y-maze test (MYM)

A modified version of the Y-maze test [25] was used as previously described [26]. The apparatus used for the MYM test was equivalent to the one used in the original Y-maze test and it consisted of black polypropylene walls with 3 arms each 40 cm long, 12 cm wide at the top, 3 cm wide at the white bottom, and 18 cm high. This test was a two-trial task with a sample phase trial and a test phase trial that were separated by an inter-trial interval (Figure 3A). In the sample phase trial, each mouse was individually placed in the maze with one of the 3 arms closed. The animals were allowed to explore the other 2 arms freely for 10 min. Test phase trial was conducted 30 min after the sample phase trial. In the test phase trial, the animal was again placed in the maze with all 3 arms opened, and allowed to explore the arms freely. In the test phase trial performed 30 min after the sample phase trial, the closed arm that was opened in the test phase trial was defined as the new arm. The arms and bottom were cleaned using 75% ethanol between trials to prevent a build-up of olfactory cues. The animal behavior was video-recorded for later analysis. Percent time spent in the new arm and numbers of total arm entries were analyzed using the SMART® ver. 2.5 system (PanLab, S.L., Barcelona, Spain).

**Figure 3:** **Diabetes-induced spatial working memory deficit in the MYM test and its reversal by test drugs.A**) Schematic drawings of the Y-maze and the experimental procedure. The maze was surrounded by different spatial cues. **A**) Experimental protocol of the MYM test. The sample trial and test trials were conducted for 5 min at a 30-min interval. (**B**) Each test was conducted 30 min (THA) or 60 min after daily oral (CTS) or i.p. (THA) administration of test drugs. % Time spent in a novel arm (B) and total locomotion distance during a 5-min observation period were analyzed. Each data column represents the mean ± S.D. (n = 6–9). #*P <* 0.05 and ###*P <* 0.001 compared with vehicle-treated *m/m* group. *P < 0.05 compared with vehicle-treated *db/db* group (Tukey test).

#### Morris water maze test (MWM)

The MWM test was performed by slightly modifying the protocol adopted in previous studies [5]. Briefly, the MWM took place during the first half of the light phase. The test was performed in a circular pool (110 cm diameter, height 30 cm) filled with water made opaque with non-fat milk and maintained at 26 ± 1°C and a circular escape platform (11 cm diameter) was submerged 1 cm below the water surface. Cues were hung at four locations at the north, west, south, and east corners of the swimming pool wall. In the first days, the animals were subjected to a visible trial (Visible 1) of the water maze in which the platform was made visible 1 cm above the water surface. Training trials were performed daily for 5 days 1 day after the visible trial. Mice received 3 trials per day as training trials. Each trial lasted until the animal found the platform, or for a maximum observation period of 120 sec for *m/m* and *db/db* groups; animals that failed to find the platform within the maximum observation period were guided there by the experimenter. In each trial, they were placed into the pool, facing the wall, with start locations varied pseudo-randomly. One day after the last acquisition training session, animals were tested in a single 120-sec probe trial without the platform. For each trial, the latency to reach the platform (escape latency), moved distance, and mean swim speed were recorded via video capture and image analysis using the SMART® system (PanLab, S.L., Barcelona, Spain).

#### Elevated plus maze test (EPM)

The EPM test was conducted by slightly modifying the protocol described in our previous reports [20,21]. Briefly, the EPM was comprised of two open arms (22 × 8 cm) and two arms enclosed by high walls (22 × 8 × 17 cm), with an open roof, the two arms of each type being positioned opposite to each other as previously described. The maze was set 60 cm above the floor. Each mouse was individually placed at the center of the maze facing one of the enclosed arms and allowed to explore the maze freely during a 10-min observation period. In this experiment, diazepam (1 mg/kg) was used as a standard anxiolytic drug and was administered intraperitoneally to the age-matched naïve db/db mice 30 min before the test. Maze performance was video-recorded for later analysis. Time spent in open arms and total locomotion distance in the maze were analyzed as indices of emotional behavior using the SMART® system (PanLab, S.L., Barcelona, Spain).

### Western blot analysis

Western blotting was performed by a slightly modified version of a method described previously [5,20,21,26]. Briefly, hippocampal tissues were dissected from the brain and proteins were extracted by homogenization in protein lysis buffer (50 mM Tris (pH 7.4), 150 mM NaCl, 0.5% sodium deoxycholate, 1%(v/v) NP-40, 0.1%(v/v) sodium dodecyl sulfate (SDS), 150 mM NaF, 8.12 μg/ml aprotinin, 2 mM sodium orthovanadate, 10 μg/ml leupeptin, and 2 mM phenylmethylsulfonyl fluoride using TissueLyser® (Qiagen, Osaka, Japan). Lysate samples were centrifuged at 10,000 rpm (4°C) for 5 min, and the supernatants were centrifuged for protein concentration assay. The protein concentration was determined using a BCA™ protein assay kit (Thermo Scientific, Rockford, IL, U.S.A.) and a microplate reader (Sunrise Classic; TECAN Japan, Kawasaki, Japan). Total protein (15 μg) prepared from each sample was electrophoresed on 7.5% SDS-polyacrylamide gel and then electro-blotted onto a polyvinylidene difluoride membrane (Clear Blot Membrane-p; ATTO). The membranes were incubated in a 5% non-fat milk-containing wash buffer (50 mM Tris (pH 7.5), 150 mM sodium chloride, and 0.1% Tween 20) for 1 h at room temperature. They were then probed with a specific antibody of interest at 4°C for 24 h. After the membranes were rinsed in TBS-T, the blots were incubated with bovine anti-goat IgG secondary antibodies linked with horseradish peroxidase (Santa Cruz Biotechnology, CA, USA) or anti-rabbit or anti-mouse secondary antibodies linked with horseradish peroxidase (DakoCytomation EnVision + System-HRP-labeled Polymer) (Dako Cytomation, Inc., Carpinteria, CA, USA) according to the manufacturer’s instructions. The immune complexes were detected by the enhanced chemiluminescence method (Immobilon® Western Chemiluminescent HRP Substrate) (Millipore, Temecula, CA, USA) and imaged using Lumino Image Analyzer LAS-4000 (Fujifilm, Tokyo, Japan). Band images were analyzed by VH-H1A5 software (Keyence, Osaka, Japan). The quantity of immunoreactive bands was normalized by comparing with their expression levels in treatment-naïve control mice. The dilution ratios and commercial sources of the antibodies used were as follows: anti-choline acetyltransferase (ChAT) goat polyclonal antibody (AB-144P; 1:3000 dilution) (Millipore, CA, USA); anti-β-actin mouse monoclonal antibody (ab8226; 1:10,000 dilution) and anti-PDGFR-α rabbit polyclonal antibody (ab61219; 1:500 dilution) (Abcam, Tokyo, Japan); anti-Akt (pan) (C67E7) rabbit monoclonal antibody (#4691; 1:1000 dilution), anti-PDGFR-β (28E1) rabbit monoclonal antibody (#3169; 1:500 dilution), anti-phospho-Akt (Ser473) rabbit polyclonal antibody (#4060; 1:500 dilution), anti-phospho-PKCα/βII (Thr638/641) rabbit polyclonal antibody (#9375; 1:1000 dilution), anti-PKCα (C67E7) rabbit polyclonal antibody (#2056; 1:1000 dilution) (Cell Signaling Technology, Danvers, MA, USA); anti-muscarinic ACh receptor rabbit polyclonal antibodies (1:500 dilution) (M1: sc-9106; M3: sc-9108; M5: sc-9106), anti-PDGF-A (E-10) mouse monoclonal antibody (sc-9974; 1:1000 dilution), anti-PDGF-B (H-55) rabbit polyclonal antibody (sc-7878; 1:1000 dilution), and anti-VEGF (A-20) rabbit polyclonal antibody (sc-152; 1:1000 dilution), (Santa Cruz Biotechnology, Santa Cruz, CA, USA); and anti-VEGFR2 rabbit polyclonal antibody (Ab-951; 1:500 dilution) (Signalway Antibody, USA).

### Immunohistochemistry

CTS administration-induced changes in expression levels of ChAT in the medial septum and VEGF in the retia of *m/m* and *db/db* mice were also examined by immunohistochemical analysis [5]. Mice were fixed by intracardiac perfusion with 4% paraformaldehyde in phosphate-buffered saline (PBS) under anesthesia. Brain and retinal tissues were post-fixed with 4% paraformaldehyde overnight at 4°C. A series of 5 μm sections were obtained by using a sliding microtome (IVS-410, SAKURA Finetek Japan, Tokyo, Japan). The paraffin-embedded specimens were deparaffinized in xylene and dehydrated with ethanol. Endogenous peroxidase was blocked with 0.1% hydrogen peroxide-methanol for 30 minutes at room temperature. Washed with Tris-buffered saline (TBS), the specimens were incubated in a microwave oven (250 W, 4 s on and 3 s off, MI-77, Azumaya, Tokyo, Japan) in target retrieval solution (Dako, Denmark) for 15 minutes and then washed with distilled water and TBS. Nonspecific binding was blocked by treatment with a special blocking reagent (Dako, Denmark) for 15 minutes. For staining of ChAT positive cells in the medial septum, the specimens were challenged with 1:400 dilution of goat anti-ChAT polyclonal antibody (AB-144P: Millipore, CA, USA) and then incubated in a moist box at 4°C overnight. Washed with TBS, the specimens were incubated with a peroxidase-conjugated bovine anti-goat IgG (Santa Cruz Biotechnology, Santa Cruz, CA, USA). After three washes in TBS, a reaction product was detected with 3,3’-diaminobenzidine tetrahydrochloride (0.25 mg/ml) and hydrogen peroxide solution (0.01%). Counter-stained with hematoxylin, the sections were rinsed, dehydrated and covered. Also included in each staining run were negative controls in which the primary antibody was omitted. The images were captured with a microscope (AX-80, Olympus, Japan). For staining of VEGF positive cells in the retina, the specimens were challenged with 1:400 dilution of anti-rabbit VEGF (A-20) polyclonal antibody (sc-152: Santa Cruz Biotechnology, Santa Cruz, CA, USA) in target retrieval solution (Dako, Denmark), incubated in a microwave oven (250 W, 4 s on and 3 s off, MI-77, Azumaya, Tokyo, Japan) for 15 minutes, and then incubated in a moist box at 4°C overnight. After washing the specimens with TBS, they were incubated with Alexa Fluor®488-conjugated goat anti-rabbit IgG antibodies (A11008; 1:400 dilution, Invitrogen, Tokyo, Japan) for 30 min at room temperature. Fluorescent images were captured using a fluorescent microscope (AX-80, Olympus, Tokyo, Japan).

### Statistical analysis

Statistical analysis of the data was conducted according to Curran-Everett and Benos [27]. All data are expressed as the mean ± S.D. The behavioral data were analyzed using paired Student’s *t*-test or one-way repeated measure ANOVA or two-way repeated measure ANOVA followed by the Tukey test for multiple comparisons among different groups. The neurochemical data were compared using unpaired Student’s *t*-test or one-way ANOVA followed by the Tukey test for multiple comparisons. Differences of *P* < 0.05 were considered significant.

## Results

### Behavioral studies

#### CTS- and THA-induced amelioration of non-spatial cognitive deficits of db/db mice in ORT

We first evaluated the non-spatial cognitive performance of *db/db* mice using the ORT, which assesses short-term memory as indicated by exploration time. Analysis of performance in the sample phase trial of the ORT revealed no differences in total time exploring two objects between each group of *m/m* and *db/db* mice [t = 0.951, df = 15, *P =* 0.356, *t*-test] [F(3, 23) = 1.914, *P =* 0.156, one-way ANOVA] (Figure 2B). These results role out the possibility that a diabetic state caused deficits of motivation and sensory motor function. However, in the test phase trial conducted 30 min after the sample phase trial, the *m/m* mice spent a significantly longer time exploring a new object than exploring a familiar object [t = -5.325, df = 7, *P =* 0.001, paired *t*-test] and exhibited a clear preference for the novel object, whereas *db/db* mice did not show a significant difference [t = 0.816, df = 8, *P =* 0.438, paired *t*-test]. On the other hand, *db/db* mice treated with CTS (750 mg/kg per day, p.o.) and THA (2.5 mg/kg per day, p.o) spent significantly longer exploring the novel object than exploring a familiar object [CTS: t = -3.643, df = 5, *P =* 0.015, paired *t*-test and THA: t = -5.765, df = 5, *P =* 0.002, paired *t*-test] (Figure 2C). These data demonstrated that vehicle-treated *db/db* mice failed to discriminate a novel object (vs. m/m group: t = 2.960, df = 15, P = 0.01, *t*-test), whereas CTS- and THA-treated *db/db* mice were clearly able to discriminate the two objects. In fact, the post hoc analysis following one-way ANOVA [F(3,23) = 4.062, *P =* 0.019] revealed that the CTS- and THA-treated *db/db* groups had a DI significantly higher than the vehicle-treated *db/db* group (Figure 2D).

#### Effect of CTS on working memory performance of db/db mice in the MYM test

A MYM test was used to evaluate the effect of CTS on spatial working memory in *db/db* animals. As shown in Figure 3, the ratio of the time that vehicle-treated control mice spent visiting the novel arm to the time spent visiting the other two familiar arms was significantly higher than the chance level of 33.3%, indicating a preference for the novel arm over the familiar arms. The vehicle-treated *db/db* mice spent significantly shorter time exploring the novel arm than the *m/m* mice [t = 4.175, df = 15, *P =* 0.001, *t*-test]. In contrast, the *db/db* mice treated with CTS and THA spent significantly longer time exploring the novel arm than the vehicle-treated group [drug treatment of *db/db* groups: F(3,23) = 4.224, *P =* 0.016; vehicle group vs. CTS 375 mg/kg per day group, *P =* 0.058; vehicle group vs. CTS 750 mg/kg per day group, *P =* 0.046; vehicle group vs. THA 2.5 mg/kg per day group, *P =* 0.017, one-way ANOVA] (Figure 3B). Locomotor activity of animals measured as total distance in the MYM test was significantly shorter in the *db/db* mice than in the *m/m* mice [t = 3.647, df = 15, *P =* 0.002, *t*-test], but the activity of *db/db* mice was not significantly affected by CTS or THA administration [F_drug_ (3,23) = 2.275, *P =* 0.107, one-way ANOVA] (Figure 3C).

#### Effect of CTS on spatial learning and memory performance of db/db mice in the MWM test

Consistent with our previous report [5], *db/db* mice showed significantly impaired spatial learning and memory performance in the MWM test. In the visible trial conducted on the first day, there was no significant difference in the time spent finding the platform between the two groups, eliminating the possibility of motivational or sensory motor deficits. The vehicle-treated *m/m* and *db/db* groups could learn the location of the submerged platform following repeated daily training [F_training_ (4,60) = 17.702, *P <* 0.001, two-way repeated measure ANOVA] (Figure 4-A1), but there was a significant difference in learning performance between two animal groups [F_animal_ (1,15) = 115.04 *P <* 0.001, two-way repeated measures ANOVA]. The escape latency of the control *db/db* group was significantly greater than that of the control *m/m* group [F_animal_ _×_ _training_ (4,60) = 5.385, *P <* 0.001, two-way repeated measure ANOVA]. Additionally, the control *db/db* mice group displayed significantly longer swimming distance to find the platform [F_distance_(1,15) = 45.604, *P <* 0.001, two-way repeated measure ANOVA] (data not shown) and swimming speed to find the platform [F_animal_(1,15) = 115.019, *P <* 0.001, two-way repeated measures ANOVA] in the training trials (Figure 4-A2). These findings indicate that *db/db* mice had not only learning and memory dysfunction but also motor dysfunction.

**Figure 4:** **Effects of CTS and THA on water maze performance of *db/db *mice.** Learning performance of the animals was analyzed in the training test by latency (**A**) and swimming speed (**B**). Each data point indicates the mean ± S.D. for 6 – 9 animals in each group. ^###^*P <* 0.001 vs. vehicle-treated *m/m* group, and ^**^P < 0.01 vs. vehicle-treated *db/db* group (one-way repeated measures ANOVA). Memory retrieval performance (D) elucidated in the probe test. Each datum represents the mean of time spent in the target quadrant ± S.D. ^###^*P <* 0.001 vs. vehicle-treated *m/m* group (*t*-test). ^*^P < 0.05 vs. respective vehicle-treated *db/db* group (one-way repeated measure ANOVA followed by Tukey test).

We also examined the effect of CTS and THA on spatial cognitive performance of *db/db* mice in the MWM test. The ameliorating effects of THA (2.5 mg/kg per day, i.p.) treatment significantly improved the reduced escape latency during the observation period in the *db/db* animal group [F_drug_ (1,13) = 17.841 P < 0.001, two-way repeated measure ANOVA] [F_training_(4,52) = 15.498, *P <* 0.001, two-way repeated measure ANOVA] [F_drug_ _×_ _training_(4,52) = 3.591, *P =* 0.012, two-way repeated measure ANOVA] and swimming distance to find the platform [F_drug_ (1,13) = 27.296, *P <* 0.001, two-way repeated measure ANOVA] in the training tests (Figure 4-A1) without affecting the swimming speed of this animal group [F_drug_ (1,13) = 2.942, *P =* 0.11, two-way repeated measure ANOVA] (Figure 4-A2). Interestingly, daily treatment of *db/db* mice with 750 mg/kg CTS also resulted in a significant decrease in escape latencies of these animal groups [F_drug_ (1,13) = 34.729, *P <* 0.001, two-way repeated measure ANOVA](Figure 4-a1), and [F_drug_ (4,52) = 8.073, *P <* 0.001, two-way repeated measure ANOVA] swimming distance [F_drug_ (1,13) = 110.616, *P <* 0.001, two-way repeated measure ANOVA] (data not shown), while CTS administration had no effect on swimming speed of *db/db* animal groups [F_drug_ (1,13) = 2.355, *P =* 0.149, two-way repeated measure ANOVA] (Figure 4-A2). In addition, CTS 375 mg/kg per day administration led to no significant changes in the training [F_drug_ (1,13) = 1.31, *P =* 0.273, two-way repeated measure ANOVA] [F_training_ (4,52) = 5.711, *P <* 0.001, two-way repeated measure ANOVA] [F_drug_ (1,13) = 0.132, *P =* 0.722, two-way repeated measure ANOVA], in the swimming distance (data not shown) and swimming speed [F_drug_ (1,13) = 0.599, *P =* 0.453, two-way repeated measure ANOVA] (Figure 4-A2).

In the probe test conducted 1 day after the 5-day training period, swimming time of the *db/db* control mice in the target quadrant where the platform had been located during training was significantly shorter than that of the *m/m* mice [t = 6.682, df = 15, *P <* 0.001, *t*-test]. The *db/db* groups treated with daily administration of CTS (375 – 750 mg/kg per day and THA (2.5 mg/kg per day) spent significantly more time in the target quadrant during the observation period than *db/db* mice treated with vehicle [F_drug_ (3,23) =14.231, *P <* 0.001, one-way ANOVA] (Figure 4C).

#### Effect of CTS on emotional performance of db/db mice in EPM test

The EPM test was conducted to evaluate the effect of CTS on anxiety-related behavior of *db/db* mice by using diazepam as a reference anxiolytic drug. The vehicle-treated *db/db* mice showed significantly decreased percentage of time spent in open arms during a 10-min observation period compared with the *m/m* controls (t = 5.082, df = 15, *P <* 0.001, *t*-test) (Figure 5A). In contrast, drug treatment of *db/db* mice significantly altered EPM behavior [F_drug_ (3,23) = 3.302, *P =* 0.0038, one-way ANOVA]. In fact, the *db/db* mice that acutely received a single dose of 1.0 mg/kg diazepam before the test spent significantly more time in the open arms than the vehicle-treated *db/db* mice. The CTS-treated *db/db* mice also spent slightly but significantly longer in the open arms than the vehicle-treated *db/db* group (Figure 5A), whereas THA treatment had no effect on the emotional performance of db/db mice. The total locomotion distance in the maze was significantly less in the vehicle-treated *db/db* mice than in the vehicle-treated *m/m* mice [t = 9.119, df = 15, *P =* 0.001, *t*-test], but the decrease of locomotor activity of the *db/db* mice was not affected by the drug administration [F_drug_ (3,23) = 0.2935, *P =* 0.830, one-way ANOVA] (Figure 5C). Indeed, total locomotion distances and swimming speeds of this diabetic animal model in MYT and WMT, respectively, were about 50% less than those of the *m/m*.

**Figure 5:** **Effects of CTS administration on EPM performance of *db/db *mice.** The animals received an **EPM** test at around the age of 13 weeks old. The 7-week-old *db/db* mice were orally administered water (vehicle), 375 – 750 mg/kg CTS, 2.5 mg/kg THA once daily during the experimental period. The EMT was conducted 1 hr after CTS administration. The age-matched naïve *db/db* mice received i.p. injection of 1 mg/kg diazepam 30 min before the test. Each datum represents the mean ± S.D. (6 – 9 animals per group). The proportion of time spent in open arms (**A**) and the total locomotion distance on the maze (**B**) were calculated. The data are expressed as the mean ± S.D. ###*P <* 0.001 vs. vehicle-treated *m/m* group (Student’s *t*-test). *P < 0.05, **P < 0.01 vs. vehicle-treated *db/db* group (one-way ANOVA followed by Tukey test).

### Biochemical studies

#### Effects of CTS and THA on serum glucose in diabetic db/db mice

Body weights and serum glucose levels of each animal group were measured before and after completion of the behavioral assessments. As summarized in Table 1, both body weights and glucose levels were significantly higher in the *db/db* mice than those in the age-matched *m/m* non-diabetic control mice. THA (2.5 mg/kg per day, i.p.) or CTS (375 – 700 mg/kg per day, p.o.) had no effect on these parameters of *db/db* mice.

**Table 1:** **Effect of CTS and THA treatment on body weight and serum glucose level in *db/db *mice**

	**7 weeks old**		**14 weeks old**				
	**m/m**	**db/db**	**m/m**	**db/db**			
			**Vehicle**	**Vehicle**	**CTS (375)**	**CTS (750)**	**THA (2.5)**
Body weight (g)	20.6 ±0.8	36.5 ±1.5	23.8 ±0.7	44.7 ±2.2	44.5 ±2.8	45.1 ±2.3	44.5 ±2.1
Serum glucose (mg/dl)	132.4 ± 9.3	281.5 ± 73.8	151.7 ±6.3	487.5. ±107.4#	420.8 ± 140.9	541.0 ± 144.9	489.4 ± 67.1

Body weights and serum glucose levels were first measured at the age of 7 weeks old just before starting drug administration. The *db/db* mice were randomly separated into 4 groups and underwent daily administration of vehicle, 375 mg/kg and 750 mg/kg CTS, or 2.5 mg/kg THA. After completion of the behavioral study, the body weight and serum glucose levels of each animal were again measured at the age of 14 weeks old. CTS and THA represent chotosan extract and tacrine, respectively. Each datum represents the mean ± S.D. (n = 6 – 9). ### *P* < 0.001 vs. respective 7w-*m/m* or 14w-*m/m* group (*t*-test).

#### Reduced AKT phosphorylation and increased PKCα phosphorylation in the db/db mice are reversed by CTS and THA administration

To understand the molecular mechanism(s) underlying CTS-induced improvement of cognitive deficits in *db/db* mice, we first examined the effects of CTS on type 2 diabetes-related AKT and PKC signaling by measuring unphosphorylated and phosphorylated levels of AKT and PKCα in the hippocampus (Figure 6). No differences in the hippocampal AKT and PKCα levels were found between the vehicle-treated *m/m* and *db/db* mice (Akt: t = 0.590, df = 8, *P =* 0.571; PKCα: t = -0.902, df = 8, *P =* 0.394), whereas the expression levels of phosphorylated AKT and PKCα in the control *db/db* group were significantly decreased (p-Akt: t = 4.690, df = 8, *P =* 0.002) and increased (p-PKCα/βII: t = -7.179, df = 8, *P <* 0.001), respectively, compared with the levels in the vehicle-treated *m/m* mice. Neither CTS nor THA treatment had any effect on the expression levels of these signaling factors in the *db/db* mice. On the other hand, repeated administration of CTS and THA significantly increased the level of p-AKT [F_drug_ (3,16) = 17.996, *P <* 0.001, one-way ANOVA] and decreased the level of phosphorylated PKCα/βII [F_drug_ (3,16) = 7.624, *P <* 0.002, one-way ANOVA] in *db/db* mice (Figure 6). No significant difference in β-actin expression in the hippocampus was observed between vehicle-treated *m/m* and *db/db* groups (t = 1.629, df = 8, *P =* 0.142). No effect of CTS or THA was found in terms of the β-actin level in the hippocampus [F_drug_ (3,16) = 0.608, *P =* 0.620, one-way ANOVA].

**Figure 6:** **Effects of CTS and THA treatment on Akt, p-Akt, PKCα, p-PKCα/βII, and β-actin in the hippocampi of *db/db *mice.** After completing the behavioral studies, the animals were decapitated and proteins were extracted from the hippocampi in each animal group. **A**) Typical photos indicating the expression levels of each factor in the hippocampus of vehicle-treated *m/m* (lane a), and vehicle (lane b)-, CTS (325 mg/kg per day: lane c; 750 mg/kg per day: lane d)-, and THA (2.5 mg/kg per day; lane e)-treated *db/db* mice. **B**) Quantitative comparisons of test drug-induced changes in Akt, p-Akt, PKCα, p-PKCα/βII, and β-actin in the hippocampi of *db/db* mice. The data are expressed as the percentage of the value obtained from naïve control *m/m* mice. Each data column represents the mean ± S.D. obtained from 5-6 brain samples. #*P <* 0.05 or ##*P <* 0.01 vs. vehicle-treated SAMR1 group (Student’s *t*-test). ##*P <* 0.01, *P < 0.05, ***P < 0.001 vs. respective vehicle-treated *db/db* group (one-way ANOVA followed by Tukey test).

#### Effects of CTS and THA on the hippocampal expression levels of VEGF and PDGF and their receptors in db/db mice

Since the VEGF/PDGF systems have been shown to play angiogenic and neurotrophic roles in the central nervous system and their function declines with aging [28-30], we evaluated the effects of the CTS treatment on the hippocampal VEGF/VEGFR2 and PDGF/PDGFR systems in *db/db* mice. Western blotting analysis (Figure 7) revealed that, compared with the vehicle-treated *m/m* mice, the vehicle-treated *db/db* mice showed reduced levels of VEGF-A (t = 3.881, df = 8, *P =* 0.005, *t*-test), VEGFR2 (t = 3.233, df = 8, *P =* 0.012, *t*-test), PDGFR-α (t = 2.855, df = 8, *P =* 0.021, *t*-test), PDGF-B (t = 4.703, df = 10, *P =* 0.002, *t*-test), and PDGFR-β (t = 3.541, df = 8, *P =* 0.008, *t*-test). The level of PDGF-A also showed a tendency to be lower in the *db/db* group than in the *m/m* group but the difference between the two groups was insignificant (t = 1.793, df = 8, *P =* 0.111, *t*-test). The CTS and THA administrations significantly up-regulated the expression levels of VEGF-A [F_drug_ (3,16) = 9.998, *P <* 0.001, one-way ANOVA], VEGFR2 [F_drug_ (3,16) = 5.267, *P =* 0.01, one-way ANOVA], PDGF-B [F_drug_ (3,20) = 4.233, *P =* 0.018, one-way ANOVA], and PDGFRβ [F_drug_ (3,16) = 7.898, *P =* 0.002, one-way ANOVA] in the *db/db* group. These drug treatments failed to reverse the down-regulated expression of PDGFRα in the *db/db* mice [F_drug_ (3,16) = 0.831, *P =* 0.496, one-way ANOVA].

**Figure 7:** **Effects of CTS and THA on VEGF/VEGFR2 and PDGF/PDGFR expression in the hippocampus of *db/db *mouse.A**) Typical photos indicating the expression levels of each factor in the hippocampus of vehicle-treated *m/m* (lane a), and vehicle (lane b)-, CTS (325 mg/kg per day: lane c; 750 mg/kg per day: lane d)-, and THA (2.5 mg/kg per day; lane e)-treated *db/db* mice. **B**) Quantitative comparisons of each factor among different animal groups were conducted as described in the text. The data are expressed as the percentage of the value obtained from naïve control *m/m* mice. Each data column represents the mean ± S.D. obtained from 5 – 6 brain samples. #*P <* 0.05, ##*P <* 0.01 vs. vehicle-treated *m/m* group (Student’s *t*-test). *P < 0.05, **P < 0.01, ***P < 0.001 vs. respective vehicle-treated *db/db* group (one-way ANOVA followed by Tukey test).

Immuno-histochemical analysis was also conducted to know whether CTS and THA treatments alter the expression level of VEGF in the retinal tissue of *db/db* mice since VEGF has been implicated as a major contributor to the development of diabetic complications such as diabetic retinopathy [31,32]. As shown in Figure 8, VEGF-positive cells were clearly observed in pigment epithelium and inner segment layers. Diabetic *db/db* mice exhibited hyperplasia in inner and outer nuclear layers, inner segments, and outer plexiform layers. They also showed increased expression of VEGF, particularly in inner segments and outer plexiform layers. However, no clear difference in the retinal morphology or the VEGF staining level was observed between vehicle-treated groups and CTS- or THA-treated *db/db* groups.

**Figure 8:** **Effects of CTS and THA on VEGF expression in the retinal tissue in *db/db *mice.** The retinal tissues were obtained from the animals perfused with paraformaldehyde as described in the text. The arrows a, b, c, and d represent pigment epithelium, outer segments, inner segments, and outer plexiform layers, respectively. VEGF-positive portions were identified by VEGF immunostaining. Photos 1, 2, 3, and 4 were from the retinal tissues of m/m control, vehicle-treated *db/db*, CTS (750 mg/kg per day)-treated *db/db*, and THA (2.5 mg/kg per day)-treated *db/db* group, respectively. Arrows a, b, c, and d represent pigment epithelium, outer segments, inner segments, and outer plexiform layer, respectively.

#### Effects of CTS and THA on downregulated expression of hippocampal cholinergic marker proteins in db/db mice

Since the central cholinergic systems play an important role in learning and memory function, we next evaluated the effects of CTS and THA treatment on the expression levels of cholinergic marker proteins in the hippocampi of *db/db* mice. Western blotting analysis (Figure 9) revealed that, compared with the control *m/m* mice, the vehicle-treated *dbdb* group had significantly reduced levels of ChAT (t = 5.074, df = 8, *P <* 0.001, *t*-test), M_1_ AChR (t = 4.951, df = 8, *P =* 0.002, *t*-test), M_3_ AChR (t = 11.128, df = 8, *P <* 0.001, *t*-test), and M_5_ AChR (t = 8.076, df = 8, *P <* 0.001, *t*-test). However, administrations of CT and THA significantly up-regulated the expression levels of ChAT [F_drug_ (3,16) = 12.379, *P <* 0.001, one-way ANOVA], M_1_ AChR [F_drug_ (3,16) = 8.689, *P =* 0.001, one-way ANOVA], M_3_ AChR [F_drug_ (3,16) = 11.943, *P <* 0.001, one-way ANOVA], and M_5_ AChR [F_drug_ (3,16) = 8.887, *P =* 0.001, one-way ANOVA] in *db/db* groups.

**Figure 9:** **Effects of CTS and THA on ChAT, M**_**1**_**, M**_**3,**_**and M**_**5**_**receptor protein expression in the hippocampus of *db/db *mouse.** Typical photos indicating the expression levels of each factor in the hippocampus of vehicle-treated *m/m* (lane a), and vehicle (lane b)-, CTS (325 mg/kg per day: lane c; 750 mg/kg per day: lane d)-, and THA (2.5 mg/kg per day; lane e)-treated *db/db* mice. B) Quantitative comparisons of each factor among different animal groups were conducted as described in the text. The data are expressed as the percentage of the value obtained from naïve control *m/m* mice. Each data column represents the mean ± S.D. obtained from 5-6 brain samples. ##*P <* 0.01, ###*P <* 0.01 vs. vehicle-treated *m/m* group (Student’s *t*-test). **P < 0.01, ***P < 0.001 vs. respective vehicle-treated *db/db* group (one-way ANOVA followed by Tukey test).

#### Immunohistochemical examination of effects of CTS and THA on septal cholinergic cells in db/db mice

Our previous report indicated that 19-week-old *db/db* mice had a significantly lower number of cholinergic cells in the medial septum and basal forebrain than age-matched *m/m* mice and 19-week-old *db/db* mice, suggesting diabetes-induced degeneration of central cholinergic systems. To understand the mechanism by which CTS treatment reverses diabetes-induced decrease of cholinergic marker proteins in the hippocampus, we immunohistochemically analyzed ChAT-immunopositive neurons in the medial septum that mainly project to the hippocampal area. Consistent with previous findings [5], the vehicle-treated *db/db* mice showed a smaller number of ChAT-immunopositive cells in the medial septum than the vehicle-treated *m/m* mice (Figure 10). The *db/db* mice administered with CTS and THA for the experimental period had a level of ChAT-immunopositive cells similar to that in the control *m/m* mice.

**Figure 10:** **Effects of CTS and THA treatment on diabetes-induced cholinergic neuron degeneration in the medial septum.** Cholinergic neurons were identified by ChAT immunostaining in vehicle-treated *m/m* (1), and vehicle (2)-, CTS (750 mg/kg per day: 3)-, and THA (2.5 mg/kg per day; 4)-treated *db/db* mice. Cholinergic neurons were stained with anti-ChAT antibody, showing that predominant ChAT expression occurred in the cell body of cholinergic neurons. Scale bar = 100 μm.

## Discussion

This study was conducted to investigate if CTS has an ameliorative effect on cognitive deficits observed in *db/db* mice as one of the diabetes-related neuropsychiatric symptoms. The results demonstrate that this type 2 diabetes animal model exhibits severe cognitive deficits, anxiety-like emotional behavior, degeneration of the basal forebrain cholinergic complexes, and down-regulation of Akt signaling and VEGF/PDGF systems in the brain and that CTS is capable of attenuating these behavioral and neurobiological deficits. Our findings suggest that CTS exhibits beneficial effects on diabetes-induced cognitive and emotional deficits and that its effects on cognitive deficits are mediated by attenuating diabetes-induced dysfunction of central cholinergic systems, and Akt signaling and VEGF/PDGF systems in the brain.

### Ameliorative effects of CTS on diabetes-induced neuropsychiatric symptoms

In this study, three different types of behavioral tasks, namely, ORT, MYT, and WMT, were used to elucidate non-spatial short-term memory [13,21], novelty-related spatial working memory [25,26], and hippocampus-dependent spatial learning and reference memory [12,33], respectively, in diabetic db/db mice and non-diabetic m/m mice. The results revealed that, compared with non-diabetic control mice, diabetic mice exhibited clearly impaired cognitive learning and memory performance in these behavioral tasks. Moreover, it was observed that diabetic mice showed reduced motor activity, that is, locomotor activity in the MYT and swimming speed in the WMT. These findings are consistent with previous reports that *db/db* mice are hypolocomotive [5,34] and have cognitive deficits [5,6,35]. Therefore, it is likely that learning and memory deficits of *db/db* mice observed in this study were caused by reduced motor activity relevant to elevated body weight of this animal group. However, this possibility seems to have been ruled out by the data obtained in our present and previous studies [5]. Indeed, our data indicated that daily administrations of THA and Kampo medicines ameliorated cognitive learning and memory performance of *db/db* mice without affecting their locomotor and swimming ability. Considering the fact that CTS and THA had no effect on serum glucose levels or body weights in *db/db* mice, these drugs likely ameliorate and/or prevent diabetes-induced cognitive deficits via a mechanism independent of anti-hyperglycemia and/or anti-obesity.

The present study also demonstrated that *db/db* mice exhibited anxiety-like behavior in the EPM test, suggesting that they are more susceptible to phobia-driven anxiety than the control *m/m* strain. This finding is in accord with the work of Dinel et al. [6]. They reported that *db/db* mice had neuropsychiatric symptoms such as cognitive deficits and anxiety-like behaviors and that the symptoms were associated with increased inflammatory cytokines and reduced expression of brain-derived neurotrophic factor (BDNF) in the hippocampus. Interestingly, in our present study, the anxiety-related behaviors of *db/db* mice were significantly attenuated in the *db/db* groups that had received an acute injection of the anxiolytic drug diazepam and daily administration of CTS. Moreover, it was of interest to note that, in contrast to CTS, THA had no effect on the emotional performance of *db/db* mice. These results suggest that CTS has a beneficial effect on neuropsychiatric symptoms of diabetic animals and allow us to speculate on possible involvement of GABAergic mechanisms in the anxiolytic-like action of CTS in *db/db* mice. However, this possibility can be ruled out for a couple of reasons. First, it is generally recognized that facilitation of central GABAergic systems by drugs such as diazepam impairs learning and memory performance [36,37]. Secondly, in our previous study using SAMP8, a senescence-accelerated mouse model, we demonstrated that repeated administration of CTS ameliorated not only cognitive deficits but also a reduced level of anxiety observed in this animal model [38]. Thirdly, there is a possibility that the anxiolytic-like effect of CTS observed in db/db mice is mediated by interaction of CTS with BNDF and VEGF/PDGF systems in the brain since these systems are reportedly implicated in attenuation of anxiety behavior in rodents [17,39]. However, considering the present and previous data obtained from THA-treated *db/db* animals, this possibility seems unlikely. THA administration failed to affect anxiety behavior of *db/db* animals, but it significantly revered the reduced levels of BDNF [5] and VEGF/PDGF in the brain. Therefore, the anxiolytic-like action of CTS may be mediated by neuronal mechanism(s) independent of central cholinergic and VEGF/PDGF systems. Further investigations are needed to clarify the mechanism(s) underlying the anxiolytic-like effect of CTS in db/db mice.

### Effects of CTS and THA on diabetes-induced neurobiological dysfunctions in the brain

We next elucidated the effects of CTS and THA administration on phosphorylation of Akt and PKCα as indices of impaired signaling and activation of PKC related to hyperglycemia-induced complications in *db/db* mice [40-42]. In this study, Akt phosphorylation and PKCα/βII autophosphorylation in the hippocampi of *db/db* mice were significantly down-regulated and up-regulated, respectively, compared with those in the control *m/m* mice and these alterations caused by diabetes were reversed by CTS and THA administrations. Evidence indicates that the Akt activation involves tyrosine kinase receptors, such as receptors for insulin, or certain growth factors, such as vascular endothelial growth factor, and that it is triggered by Akt phosphorylation via phosphatidylinositol 3 kinase and phosphoinositide-dependent protein kinases. An Akt activation mechanism is reduced in the CNS of diabetes models including *db/db* mice [43,44], although there is a report with conflicting findings [45]. Moreover, recently it was reported that phosphatidylinositol 3-kinase cascade including Akt phosphorylation is involved in neuroprotective influence of cholinergic drugs on glutamate-induced neurotoxicity [46], indicating that PI3K-Akt signaling pathway plays an important role in the cholinergic mechanism [47]. On the other hand, it is generally believed that intracellular PKC is activated by the diabetes-induced accumulation of its co-factor, diacylglycerol, inside the cells [48] and that, once activated, PKC undergoes autophosphorylation via translocation from the cytosol to the plasma membrane and other subcellular compartments [41]. Therefore, our data are consistent with these findings. Considering the effects of THA, our findings suggest that CTS and THA can improve dysfunctions of the Akt and PKC signaling systems in the CNS of diabetic *db/db* animals via facilitation of central cholinergic systems and that these effects are independent of their effects on serum glucose levels.

Interestingly, this study demonstrated that, compared with the vehicle-treated non-diabetic control group, the vehicle-treated *db/db* group exhibited down-regulation of the VEGF/PDGF signaling systems in the hippocampus that were reversible by CTS and THA administration. VEGF is a hypoxia-inducible secreted protein that interacts with receptor tyrosine kinases such as VEGFR2 on endothelial cells and promotes angiogenesis. PDGF as well as VEGF plays an important role in angiogenesis that depends on endothelial cell invasion and proliferation and requires pericytes coverage of vascular sprouts for vessel stabilization. VEGF and PDGF coordinate these processes on endothelial cells and vascular smooth muscle cells, respectively [49,50]. Moreover, these growth factors are implicated in the adverse vascular effects of hyperglycemia-related complications [15,51] and their functions in the peripheral tissues are up-regulated. Therefore, down-regulation of VEGF/VEGFR and PDGF/PDGFR systems found in this study was in contrast to these previous findings. Recent evidence indicates that the signaling pathways of VEGF and PDGF receptors also involve Akt activation via phosphatidylinositol-3 kinase/Akt pathways and thereby exhibit neuroprotective activities [52,53] or mediate protective influence of cholinergic drugs on ischemic cell damage [54,55]. Therefore, it is likely that alterations of expression levels of VEGF/PDGF and their receptors in the hippocampus are relevant to the aforementioned decrease of phosphorylated Akt in the *db/db* mice.

In the central nervous system, VEGF and VEGFR2 are expressed not only in vascular endothelial cells but also in other cells such as neurons and neural progenitor cells [56] and are involved in brain functions including enhancement of neurogenesis through the direct activation of neural progenitor cells [57], amelioration of cognitive deficits via the promotion of neurogenesis, and protection of endothelial cells and neurons during brain ischemia in adult rats [57,58]. There is also evidence that PDGF-A and -B and their receptors (PDGFRα and PDGFRβ) play a role not only in the proliferation, migration, and differentiation of oligodendrocytes [59] but also in neurite outgrowth [60] and neuroprotection via phosphatidylinositol 3-kinase, a mitogen-activated kinase kinase pathway [30]. These signaling mechanisms are important in the long-term potentiation of learning and memory, a biological index of memory formation [61]. We previously reported using a senescence-accelerated mouse model that aging induces dysfunction of the VEGF/VEGFR2 and PDGF/PDGFR signaling systems in the brain and that reversal of impaired VEGF/VEGFR2 and PDGF/PDGFR signaling systems is a part of the mechanism(s) underlying the ameliorative effects of CTS on spatial and non-spatial cognitive deficits caused by aging [20]. Taken together, the present results suggest that the CTS-induced reversal of expression level changes of VEGF/VEGFR2 and PDGF-B/PDGFRβ in *db/db* mice contributes to the improvement of cognitive performance by CTS administration.

It is of interest to note that the effects of CTS and THA on VEGF/PDGF systems in the brain of *db/db* animals were different from those on the retina in *db/db* mice. VEGF/PDGF has been implicated as a major contributor to the development of diabetic complications such as diabetic retinopathy [32,62]. Elevated expression of VEGF and its receptor has also been demonstrated in diabetic retinas [63]. These roles of VEGF/PDGF in diabetic complications raise the possibility that CTS administration may exacerbate diabetic retinopathy. However, this possibility seems to be little since, although VEGF was highly stained in the endothelial cells and microvessel regions of *db/db* mice compared with that in the control *m/m* mice are consistent with these previous reports, CTS or THA treatment had no effect on the retinal VEGF expression in the *db/db* mice. The reason for the different susceptibility of VEGF/PDGF systems to CTS and THA treatment between the brain and retinal tissues is unclear. However, there may be a difference in the mechanism to regulate expression of these factors between the central nervous system and the peripheral tissues.

### Protective effects of CTS and THA administration against dysfunction of central cholinergic systems

To obtain a better understanding of the mechanism by which CTS ameliorates cognitive deficits in *db/db* diabetic animals, we next elucidated the effect of CTS and THA on the central cholinergic systems since these systems play an important role in cognitive performance and their hypofunction is closely related to the progression of memory deficits [64,65]. Indeed, evidence indicates that muscarinic receptors such as M_1_, M_3_, and M_5_ subtypes have an important role in cognitive function in rodents [13,66-68]. In this study, we found that the expression levels of cholinergic marker proteins in the hippocampus, namely, choline acetyltransferase (ChAT) and muscarinic M_1_, M_3_, and M_5_ receptors, were down-regulated in the vehicle-treated *db/db* mice compared with those in the age-matched vehicle-treated *m/m* group and that CTS treatment, as well as THA treatment, reversed the downregulated expression of these proteins in *db/db* mice. These findings are consistent with our previous study that db/db mice had dysfunction of the central cholinergic systems [5]. In the previous study, we demonstrated that the dysfunction likely occurs in an aging-dependent manner and is accelerated in *db/db* mice because no differences in expression levels of these marker proteins were observed when compared between young (7-week-old) *db/db* mice and age-matched *m/m* mice. Taking these findings together, one of the plausible explanations for CTS- and THA-induced amelioration of cognitive deficits of *db/db* mice is that these drugs in part protect the central cholinergic systems from aging-induced degeneration of cholinergic neurons that is accelerated in *db/db* animals. This idea is supported by the present immunohistochemical study that the medial septum in *db/db* mice had fewer ChAT-immunopositive cells providing projections to the hippocampus than that in the age-matched control *m/m* mice and that the decrease of the cells was prevented in the *db/db* groups treated with CTS and THA. The reversal of downregulated expression of the cholinergic marker proteins in CTS- and THA-treated *db/db* mice seems to be consistent with the findings reported by Kakinuma et al. [54,55]. They demonstrated using cardiomyocytes that an increase in acetylcholine level by an acetylcholinesterase inhibitor or vagal nerve stimulation directly transduces cell survival signal through muscarinic receptors, activates the PI3K/Akt/HIF-1α/VEGF pathway, and leads to protection of the cell and increase of ChAT expression.

It is of interest that the effects of CTS on cognitive function and central cholinergic systems in db/db mice are quite similar to those of THA. From these findings, one may infer that chemical constituents and/or their metabolites of CTS have a potential to inhibit the activity of acetylcholinesterase in the brain; however this possibility seems to be little, since, in our previous study, administration of THA but not CTS reduced *ex vivo* activity of acetylcholinesterase in the brain [13]. Our findings suggest that the mechanism of action of CTS may differ from that of THA. Therefore, the exact mechanism underlying CTS-induced modulation of central cholinergic systems in db/db mice requires further investigations.

## Conclusion

CTS, as well as THA, attenuates cognitive deficts in *db/db* mice. The effects of CTS involve reversal of diabetes-related dysfunction of insulin signaling, down-regulation of VEGF/PDGF signaling systems, and neurodegeneration of central cholinergic systems. These findings provide further evidence for the anti-dementia effect of CTS. Moreover, this study demonstrates that CTS also has a beneficial effect on diabetes-induced emotional deficits and that the effect is likely mediated by a mechanism different from that involved in the effect on cognitive deficits.

## Abbreviations

AD: Alzheimer’s disease; CTS: Chotosan; ChAT: Choline acetyltransferase; BDNF: Brain-derived neurotrophic factor; VEGF: Vascular endothelial growth factor; VEGFR2: VEGF receptor type 2; PDGF: Platelet-derived growth factor; PDGFRα: PDGF receptor α; PDGFRβ: PDGF receptor β; 3D-HPLC: Three-dimensional high-performance liquid chromatography; LC-MS: Liquid chromatography-mass spectrometry; ESI: Electrospray ionization; ORT: Object recognition test; MYM: Modified Y-maze; MWM: Morris water maze; EPM: Elevated plus maze; TBS: Tris-buffered saline; ANOVA: Analysis of variance.

## Competing interests

The authors declare that they have no competing interests.

## Authors’ contributions

QZ, YN, KM, KET, KOT, and TY were responsible for the study concept and design. QZ and YN contributed to data acquisition, QZ, YN, KM, and TY assisted with data analysis and interpretation of findings. QZ, YN, and KM drafted the manuscript. TM provided critical revision of the manuscript. All authors read and approved the final version of the manuscript.

## Pre-publication history

The pre-publication history for this paper can be accessed here:

http://www.biomedcentral.com/1472-6882/12/188/prepub
